# The Effectiveness and Safety of Ropivacaine and Medium-Dose Dexmedetomidine in Cesarean Section

**DOI:** 10.1155/2022/4447484

**Published:** 2022-06-21

**Authors:** Bin-Bin Huang, Shi-Kun Niu

**Affiliations:** Department of Surgical Anesthesia, Shiyan Maternal and Child Health Hospital, Shiyan, China

## Abstract

*Objective*: To study the effects of epidural anesthesia with different doses of dexmedetomidine and ropivacaine on postoperative hemodynamics and neonatal outcome of cesarean section parturients. *Methods*. A total of 90 parturients who underwent cesarean section admitted to our hospital from January 2019 to January 2020 were selected as the research objects and were divided into groups A, B, and C according to different dosages of dexmedetomidine, with 30 cases in each group. Groups A, B, and C were given dexmedetomidine 0.5 *μ*g/kg, 0.8 *μ*g/kg, 1.0 *μ*g/kg, respectively, combined with 0.2% ropivacaine. The anesthesia effect, traction response, hemodynamic indexes, and neonatal Apgar score of the three groups were compared; the “Numerical Rating Scale (NRS) Score” was used to assess the postoperative pain of the parturients, and the “Ramsay Sedation Scale” was used to assess the sedation state of the parturients. *Results*. The superior anesthesia effect of group B was obtained compared with groups A and C (*P* < 0.05). Group B witnessed a lower degree of grade III stretching response, as compared to group A (*P* < 0.05). In comparison with groups A and C, superior results of the heart rate and mean artery pressure (MAP) of group B at T1 and T2 were obtained (*P* < 0.05). The neonatal Apgar score in group B was lower than those in groups A and C (*P* < 0.05), and the NRS score of group B was also lower than that of group A (*P* < 0.05). Compared with groups A and C, group B yielded a more favorable outcome in terms of the Ramsay score (*P* < 0.05). *Conclusion*. The use of medium-dose dexmedetomidine in cesarean section parturients is safer and can effectively reduce the impact on maternal hemodynamics, which is worthy of promotion and application.

## 1. Introduction

Cesarean section, as a common operation in obstetrics and gynecology, is currently widely used and an effective means to save the lives of mothers and infants [1]. With the advancement of medical technology and the improvement of living standards, people's requirements for clinical anesthesia effects and safety have become more stringent. At present, epidural anesthesia, as a common anesthesia method for cesarean section, is characterized by small impact on the fetus and an excellent controllability [2–4]. Most parturients are susceptible to a variety of factors during cesarean section, which can cause dramatic mood swings, and due to the lack of knowledge of the operation process and the unfamiliarity to relevant delivery experience, parturients who are to first experience cesarean section are also prone to anxiety, depression, and other negative emotions, which will seriously reduce the quality of delivery [5, 6]. In addition, epidural anesthesia for women undergoing second cesarean section is prone to a short duration of anesthesia block, and it is often accompanied by adverse events such as nausea and traction-related reactions during the operation. Based on this, the actual situation of the parturients should be fully assessed before performing anesthesia surgery to further stabilize their heart rate and blood pressure and relieve the negative emotions.

The most important features of pain-free delivery are pain avoidance, reduced fear of childbirth, and reduced postpartum fatigue [7]. It can also reduce unnecessary oxygen consumption, prevent maternal and infant metabolic acidosis, reduce uteroplacental blood flow, and improve fetal oxygen and condition [8]. Related studies have found that dexmedetomidine can stable hemodynamics and analgesia, improve the effect of the local anesthesia in cesarean section, and avoid the occurrence of adverse events [9–11]. In addition, ropivacaine can reduce the immune stress response of the parturients, so the combined use of the two exerts a promising clinical effect. In previous studies on the combined use of dexmedetomidine and ropivacaine, more attention was paid to the effect of the two used in epidural anesthesia, while the effects of different doses of dexmedetomidine combined with ropivacaine for epidural anesthesia on postoperative hemodynamics and the neonatal outcome of cesarean section parturients are rarely reported [12, 13]. In order to further explore the effect of different doses of dexmedetomidine and ropivacaine for epidural anesthesia on postoperative hemodynamics and the neonatal outcome of cesarean section parturients, this study matched 90 cases of parturients who underwent cesarean section in our hospital from January 2019 to January 2020 as the research objects. The results are summarized as follows.

## 2. Materials and Methods

### 2.1. General Information

A total of 90 parturients who underwent cesarean section and admitted to our hospital from January 2019 to January 2020 were selected as the research objects. They were divided into groups A, B, and C according to different doses, with 30 cases in each group.

### 2.2. Inclusion Criteria

Inclusion criteria were defined as follows: ① age >18 years old; ② all who were singleton full-term pregnancy and who met the surgical indications would go through cesarean section to end the delivery; ③ this study was approved by the hospital ethics committee, and the patients and their family members understood the purpose and process of the study and signed the informed consent.

### 2.3. Exclusion Criteria

Exclusion criteria were defined as follows: ① combined with primary hematopoietic system diseases and primary immunodeficiency diseases; ② had recently taken analgesics; and ③ with contraindications to surgery.

### 2.4. Methods

All parturients were given epidural anesthesia. Before the operation, they were fasted for 6 hours and forbidden to drink for 8 hours. The temperature of the operating room was maintained at around 24°C. In the meanwhile, the vital signs of the parturients were closely monitored. In order to prevent accidents, intravenous infusion of upper extremities should be established to prepare for first aid. Puncture method: the parturient took the left lateral decubitus position, and epidural puncture at L_2-3_ was performed to observe whether there was blood return. After the puncture, the parturient took the supine position, and 3 mL of 2% Lidocaine (Manufacturer: Chengdu First Pharmaceutical Co., Ltd.; H51021662; specification: 5 ml: 0.1 g) was injected as the test volume. After observing for 6 minutes without abnormalities and excluding signs of spinal anesthesia, group A was given intravenous infusion of 0.5 *μ*g/kg dexmedetomidine (Manufacturer: Jiangsu Hengrui Pharmaceutical Co., Ltd.; Guoyao Zhunzi H20090248; specification: 2 mL: 200 *μ*g), combined with 15 mL 0.2% ropivacaine (Manufacturer: Guangdong Jiabo Pharmaceutical Co., Ltd.; Guoyao Zhunzi H20173194; specification 20 mL: 200 mg) mixed with 2 mL physiological saline. Dexmedetomidine for group B was changed to 0.8 *μ*g/kg, and for group C, it was changed to 1.0 *μ*g/kg. The rest were the same as group A, and the infusion time for the three groups was all 15 minutes. All operations were performed by the same group of gynecologists.

### 2.5. Observation Indicators

In comparing the anesthesia effects of the three groups, if there were no adverse reactions, the induction of anesthesia was stable, and if the vital indicators were normal, it would be marked as excellent; if there was slight restlessness and the muscle relaxation was good, it would be marked as average; if the muscle relaxation was poor and accompanied by pain, then it would be marked as medium; if the anesthesia failed, and other anesthesia methods were used to complete the operation, it would be marked as bad. Effective rate = (excellent + good)/total number of cases ^*∗*^ 100%.

The time points of before the operation, 30 min during the operation, and at the end of the operation were set as T0, T1, and T2, separately. The hemodynamic indexes of the three groups at different time points were observed and compared. The hemodynamic indexes include the heart rate (HR) and mean arterial pressure (MAP).

The stretching response of the three groups was observed: grade I represented comfortable and quiet; grade II stood for the pain of stretching within a tolerable range; grade III as unbearable.

The “Apgar Score” [14] was used to evaluate the physical status of the three groups. The scale had a full score of 10 points. The lower the score, the more severe the asphyxia of the newborn.

The “NRS” [15] was used to assess the postoperative pain intensity of the parturients. The scale had a total score of 10 points. The higher the score, the more severe the pain of the parturients.

The “Ramsay Sedation Rating Scale” [16] was to evaluate the postoperative sedation status of the three groups of parturients. The total score of the scale was 6 points. The higher the score, the better the sedation effect.

### 2.6. Statistical Analysis

SPSS20.0 was selected to process the data in this study, and GraphPad Prism 7 (GraphPad Software, San Diego, USA) was used to draw the data. The study included count data and measurement data, using *x*^2^-tests, *t*-test, and the test of normality. *P* < 0.05 was considered to be statistically significant.

## 3. Results

### 3.1. Comparison of Clinical Data of the Three Groups

There were no significant differences in the age, height, body mass index (BMI), average gestational week, and residence of the three groups of parturients (*P* > 0.05), and they were comparable, as shown in Table 1.

### 3.2. Comparison of Anesthesia Effects of the Three Groups

Superior anesthesia effect of group B was obtained compared with groups A and C (*P* < 0.05), as shown in Table 2.

### 3.3. Comparison of Traction Responses of the Three Groups

Group B witnessed a lower degree of grade III stretching response, as compared to group A (*P* < 0.05), as shown in Table 3.

### 3.4. Comparison of HR of the Three Groups at Different Time Points

The heart rate at T0, T1, and T2 in group A was (88.34 ± 10.21) times/min, (85.27 ± 8.38) times/min, and (86.33 ± 10.25) times/min, respectively, while in group B, the heart rate at T0, T1, and T2 was (88.35 ± 9.35) times/min, (80.21 ± 4.25) times/min, and (81.22 ± 5.12) times/min, respectively; the heart rate at T0, T1, and T2 in group C was (88.21 ± 10.21) times/min, (94.22 ± 9.32) times/min, and (96.33 ± 11.25) times/min, respectively. In comparison with groups A and C, the heart rate of group B at T1 and T2 was lower (*P* < 0.05), as shown in Figure 1.

### 3.5. Comparison of MAP Indexes of the Three Groups at Different Time Points

The MAP indexes at T0, T1, and T2 in group A was (82.37 ± 7.32) mmHg, (87.69 ± 9.11) mmHg, and (88.35 ± 10.05) mmHg, respectively, while in group B, the MAP indexes at T0, T1, and T2 was (82.24 ± 7.41) mmHg, (83.01 ± 7.55) mmHg, and (83.27 ± 8.23) mmHg, respectively; the MAP indexes at T0, T1, and T2 in group C was (82.32 ± 7.29) mmHg, (95.33 ± 9.35) mmHg, and (97.35 ± 11.23) mmHg, respectively. In comparison with the groups A and C, the MAP index of group B was less (*P* < 0.05), as shown in Figure 2.

### 3.6. Comparison of the Apgar Score of the Three Groups

The Apgar score of group A was (9.01 ± 1.12) points; the Apgar score of group B was (8.22 ± 1.05) points; the Apgar score of group C was (9.21 ± 1.21) points. In comparison with the groups A and C, a superior outcome of the Apgar score of group B was obtained (*P* < 0.05), as shown in Figure 3.

### 3.7. Comparison of the NRS Score of the Three Groups

The NRS score of group A was (7.23 ± 1.24) points; the NRS score of group B was (4.32 ± 1.01) points; the NRS score of group C was (3.98 ± 0.96) points. In comparison with the group A, a lower score of the NRS score of group B was obtained (*P* < 0.05), as shown in Figure 4.

### 3.8. Comparison of the Ramsay Score of the Three Groups

The NRS score of group A was (2.37 ± 0.56) points; the NRS score of group B was (4.98 ± 1.23) points; the NRS score of group C was (2.41 ± 0.66) points. Compared with groups A and C, group B yielded a more favorable outcome in terms of the Ramsay score (*P* < 0.05), as shown in Figure 5.

## 4. Discussion

Pregnancy will affect maternal organ function, and the implementation of effective anesthesia in cesarean section can not only relieve maternal pain but also reduce the impact on mothers and infants [17, 18]. Compared with conventional anesthesia, epidural anesthesia with a higher maternal acceptance enjoys a rosy analgesic effect, which is widely used in clinical practice. This kind of anesthesia method is to inject local anesthetics into the epidural space of parturients, which aims to block the spinal nerve root and produce temporary analgesic anesthesia effect in the nearby area, so as to bring down the stress response of parturients [19–21]. In addition, the parturients will be in a relatively conscious state to feel the contractions in the whole process of labor. Due to the existence of risk of epidural anesthesia technology, which is easy to be affected by individual differences of the parturients, it can result in different analgesic effects and labor processes with the different dosages of anesthetics. Besides, during the operation, the parturients are prone to anxiety and other negative emotions, which excites the sympathetic nerve and dilates the uterus, thus affecting the uterine contraction, which will increase the incidence of bleeding and other adverse events, and they affect the operation results [22, 23]. The rational use of sedatives and anesthetics can ensure the comfort and safety of the parturients and reduce the harmful stimulation to them as well, so as to alleviate the pain and negative emotions, which is conducive to the prognosis.

Dexmedetomidine is a common high selective *α* 2 adrenoceptor agonists in clinical practice, which is characterized by a short action time and a strong analgesic effect, and the analgesic mechanism is through the locus ceruleus of the brain stem *α* 2 adrenergic receptors to play the role of analgesia and reduce maternal stress response. However, it is clinically found that a variety of adverse reactions may occur after using dexmedetomidine, such as dry mouth, nausea, and dizziness, which is mostly positively related to the application dose of dexmedetomidine [24, 25]. Many hospitals prescribe dexmedetomidine for use in pregnant women only when the potential benefit outweighs the potential risk to the fetus [26]. In addition, studies have shown that radioisotope-labeled dexmedetomidine is secreted in breast milk after subcutaneous administration to lactating female mice, so this product should be used with caution in lactating women [27]. As a new type of a long-acting amide local anesthetic, ropivacaine has the advantages of low toxicity and quick onset, which can promote the rapid recovery of the maternal body, so it is widely used in cesarean operations. It can inhibit the sodium ion channel of nerve cells and block the flow of sodium ions into the nerve fiber cell membrane, thereby reversibly blocking the impulse conduction along the nerve fiber. And the side effect of this drug on the motor nerve block is rather hidden, so the parturients can freely carry out activities after the operation [28]. Because it is not an intravenous anesthesia, it is a relatively safe anesthetic drug that will not pass through the blood between the mother and the fetus [29]. However, it has many disadvantages when used alone, including hypotension, excessive sedation, bradycardia, and prolonged secondary labor [30].

This study found that the heart rate and MAP indexes of group B at T1 and T2 were significantly lower than those of groups A and C (*P* < 0.05), indicating that the 0.8 *μ*g/kg dose of dexmedetomidine and 0.2% ropivacaine in epidural anesthesia could effectively reduce the hemodynamic parameters during maternal surgery, reduce the occurrence of adverse reactions during surgery, and improve the safety of the operation. Moreover, compared with groups A and C, the anesthesia effect of dexmedetomidine at a dose of 0.8 *μ*g/kg was better, which was beneficial to alleviate the negative emotions and improve the prognosis of the parturients. The results of this study showed that the Apgar score of group B was significantly lower than that of groups A and C (*P* < 0.05), which was consistent with the research results of ANNIEK F et al. [26] who pointed out that “the Apgar score of newborns in group D0.8 was (7.38 ± 1.11) points, significantly better than the (9.11 ± 0.24) points and (9.17 ± 0.58) points (*P* < 0.05) of the D0.6 group and D1.0 group (*P* < 0.05),” indicating that the 0.8 *μ*g/kg dose of dexmedetomidine has a little effect on the newborns.

After pregnancy, a woman's body loses a lot of DHA elements, which can lead to memory loss [31]. During pregnancy, many pregnant women experience pregnancy complications such as gestational hypertension and gestational diabetes, and their body's resistance to infection deteriorates after pregnancy [32]. Weakness and fatigue may occur after delivery, and joint pain may result if exposed to wind and cold [33]. According to traditional Chinese medicine, the main problem for women after childbirth is weakness of energy and blood, which is caused by the loss of blood and qi during labour [34]. The woman's body is often weak and her resistance is poor, making her susceptible to infections [35]. Postnatal care is particularly important as the postnatal period is a period of weakness and fatigue due to the depletion of blood and energy. Traditional Chinese medicine emphasizes that the mainstay of postpartum care should be to nourish the blood and replenish kidney yin [35]. Pregnant women can take Ten Perfect Tonic and Eight Precious Soup, or they can eat Astragalus and Angelica to nourish the energy and replenish the blood and add Chinese wolfberries [36].

Finally, our horizon's sample size is small, and the results may be inaccurate, affecting the results. In addition, different clinical centers, different time periods, different instruments, and different postoperative pain assessments can increase the heterogeneity of results. We need to conduct further clinical trials in multiple centers.

## 5. Conclusion

In summary, the application of medium-dose dexmedetomidine and ropivacaine in cesarean section can effectively reduce the pain of the parturients and yields a promising anesthesia effect and high safety, which is worthy of promotion and application.

## Figures and Tables

**Figure 1:** Comparison of the HR of the three groups at different time points (*x* ± *s*). The abscissa represented time of T0, T1, and T2, and the ordinate represented heart rate (times/min). ^*∗*^indicates that there was a significant difference in the heart rate of the three groups at T1 (*t* = 4.784, *P*=0.002); ^*∗∗*^indicates that there was a significant difference in the heart rate of the three groups at T1 (*t* = 4.245, *P*=0.006).

**Figure 2:** Comparison of MAP indexes of the three groups at different time points (*x* ± *s*). The abscissa represented time of T0, T1, and T2, and the ordinate represented the MAP index (mmHg). ^*∗*^indicates that there was a significant difference in the MAP index of the three groups at T1 (*t* = 3.662, *P*=0.012); ^*∗∗*^indicates that there was a significant difference in the MAP index of the three groups at T2 (*t* = 3.650, *P*=0.013).

**Figure 3:** Comparison of the Apgar score of the three groups (*x* ± *s*). The abscissa represented groups A, B, and C, and the ordinate represented the Apgar score (points). ^*∗*^indicates that there was a significant difference in the Apgar score between groups A and B (*t* = 2.818, *P*=0.007); ^*∗∗*^indicates that there was a significant difference in the Apgar score between groups B and C (*t* = 3.385, *P*=0.001).

**Figure 4:** Comparison of the NRS score of the three groups (*x* ± *s*). The abscissa represented after operation, and the ordinate represented the NRS score (points). ^*∗*^indicates that there was a significant difference in the NRS score between groups A and B (*t* = 9,966, *P* < 0.001); ^*∗∗*^indicates that there was a significant difference in the NRS score between groups A and C (*t* = 11.341, *P* < 0.001).

**Figure 5:** Comparison of the Ramsay score of the three groups (*x* ± *s*). The abscissa represented after operation, and the ordinate represented the Ramsay score (points). ^*∗*^indicates that there was a significant difference in the Ramsay score between groups A and B (*t* = 10.578, *P* < 0.001); ^*∗∗*^indicates that there was a significant difference in the NRS score between groups B and C (*t* = 10.084, *P* < 0.001).

**Table 1:** Comparison of clinical data of the three groups (*n* (%)).

	Group A (*n* = 30)	Group B (*n* = 30)	Group C (*n* = 30)	*x* ^2^/*t* value	*P* value
Age (years)				0.281	0.780
	25.37 ± 2.32	25.11 ± 2.45	25.23 ± 2.38		
Height (cm)				0.142	0.887
	1.67 ± 0.38	1.65 ± 0.35	1.66 ± 0.36		
BMI (kg/m^2^)				0.141	0.887
	27.31 ± 2.33	27.22 ± 2.45	27.35 ± 2.27		
Average gestational week (weeks)				0.248	0.805
	38.45 ± 2.33	38.22 ± 2.45	38.32 ± 2.38		
Place of residence				0.317	0.853
Urban	20 (66.67)	21 (70.00)	22 (73.33)		
Rural	10 (33.33)	9 (30.00)	8 (26.67)		

**Table 2:** Comparison of anesthesia effects of the three groups.

Group	No.	Excellent	Good	Average	Poor	Effective rate
Group A	30	50.00% (15/30)	10.00% (3/30)	13.33% (4/30)	26.67% (8/30)	73.33% (18/30)
Group B	30	66.67% (20/30)	26.67% (8/30)	6.67% (2/30)	0.00% (0/30)	93.33% (28/30)
Group C	30	53.33% (16/30)	13.33% (4/30)	10.00% (3/30)	23.33% (7/30)	66.67% (20/30)
*X* ^2^ value						9.545
*P* value						＜0.05

**Table 3:** Comparison of traction responses of the three groups (*n* (%)).

Group	No.	Grade I	Grade II	Grade III
Group A	30	36.67% (11/30)	30.00% (9/30)	33.33% (10/30)
Group B	30	66.67% (20/30)	23.33% (7/30)	10.00% (3/30)
Group C	30	63.33% (19/30)	30.00% (9/30)	6.67% (2/30)
*X* ^2^ value		5.931	0.443	4.812
*P* value		0.015	0.506	0.028

## Data Availability

The datasets used during the present study are available from the corresponding author upon reasonable request.
